The article "Long Noncoding RNA TFAP2A-AS1 Suppressed Hepatitis B Virus Replication by Modulating miR-933/HDAC11" was retracted in 2023. Reasons: unreliable results or conclusions; lack of ethics approval or compliance; concerns about the data; concerns about the peer review.

# Long Noncoding RNA TFAP2A-AS1 Suppressed Hepatitis B Virus Replication by Modulating miR-933/HDAC11

**DOI:** 10.1155/2022/7733390

**Published:** 2022-04-18

**Authors:** Yu Cheng, Weiwu Shi, Xudong Cui, Lei Sun, Yi Nan, Hong Yao, Jian Fan, LiYing Zhu, Lei Yu

**Affiliations:** ^1^Department of Infectious Disease, The Fourth Hospital of Harbin Medical University, Harbin, 150001 Heilongjiang, China; ^2^Department of integrated internal medicine, Shanghai Donghai Senior Nursing Hospital, Shanghai, China; ^3^Department of Ophthalmology, The Fourth Hospital of Harbin Medical University, Harbin, 150001 Heilongjiang, China; ^4^Traditional Chinese Medicine College of Ningxia Medical University, Yinchuan 750004, China; ^5^Department of Infectious Disease, The Second Hospital of Harbin Medical University, Harbin, 150000 Heilongjiang, China

## Abstract

**Objective:**

Studies have shown that long noncoding RNAs (lncRNAs) play crucial roles in multiple tumor types and regulate various biological processes. The present study tried to study lncRNA TFAP2A-AS1 in HBV infection hepatocellular carcinoma.

**Methods:**

The level of TFAP2A-AS1 and miR-933 in HCC cell and samples were detected by qRT-PCR assay. Luciferase reporter gene assay was carried out to study the mechanism of TFAP2A-AS1 and miR-933. Cell proliferation was measured by CCK-8 assay. HBV DNA replication was detected by RT-qPCR.

**Results:**

We firstly demonstrated that TFAP2A-AS1 was downregulated in HCC cell lines and HBV-infected HCC samples compared with nontumor tissues. However, miR-933 was upregulated in HCC cell lines and HBV-infected HCC samples compared with nontumor tissues, and miR-933 was negatively associated with the expression of TFAP2A-AS1 in HBV-correlated HCC samples. TFAP2A-AS1 and HDAC11 expression was decreased and miR-933 was upregulated in the HBV-infected cell HepG2.2.15. TFAP2A-AS1 acted as a sponge for miR-933 and HDAC11 was one direct target gene for miR-933. Overexpression of TFAP2A-AS1 suppressed cell growth, HBV DNA replication, HbeAg, and HbsAg expression, while knockdown of TFAP2A-AS1 enhanced cell proliferation, HBV DNA replication, HbeAg, and HbsAg expression in HepG2.2.15 cell. In addition, ectopic expression of miR-933 promoted cell growth, HBV DNA replication, HbeAg, and HbsAg expression in HepG2.2.15 cell. TFAP2A-AS1 suppressed HBV replication and infection through regulating HDAC11.

**Conclusion:**

These data demonstrated that TFAP2A-AS1 acted crucial roles in the modulation of HbeAg and HbsAg expression and HBV replication and may be one potential target for HBV infection treatment.

## 1. Introduction

HBV (hepatitis B virus) could cause acute or chronic infection of hepatitis B, which was supposed to be the most risk factor for hepatocellular carcinoma and chronic liver cirrhosis [1–4]. Epidemiological reports show that there are 400 million people with HBV infection worldwide and the number is still increasing. Importantly, more than 30% HBV infection cases were from China [5–7]. HBV can relax genome of rcDNA (circular DNA) in the nucleocapsid and then converted into cccDNA (covalently closed circular DNA), which acted important roles in viral persistence [8–10]. Thus, it is of great significance to investigate the mechanism of HCC development induced by HBV.

The article "Long Noncoding RNA TFAP2A-AS1 Suppressed Hepatitis B Virus Replication by Modulating miR-933/HDAC11" was retracted in 2023. Reasons: unreliable results or conclusions; lack of ethics approval or compliance; concerns about the data; concerns about the peer review.

Long noncoding RNAs (lncRNAs) are one group of transcripts more than 200 nucleotides in length that have limited or no protein-coding capacity [11–16]. References revealed that lncRNAs were misregulated in a variety of tumors including bladder tumor, ovarian cancer, neuroblastoma, gallbladder cancer, and also HBV-induced hepatocellular carcinoma [17–21]. LncRNAs regulate diverse cell processes such as cell differentiation, development, apoptosis, metabolism, and protein synthesis [22–27]. Recently, TFAP2A-AS1 has been identified to be downregulated in breast cancer cell and samples, and TFAP2A-AS1 overexpression suppressed cell invasion and proliferation and decreased tumor development in vivo [28]. However, its role in HBV infection and HBV-correlated HCC remains uncovered.

We manifested that TFAP2A-AS1 was downregulated in HCC cell lines and HBV-infected HCC samples and ectopic expression of TFAP2A-AS1 suppressed HBV replication and infection.

## 2. Materials and Methods

### 2.1. Clinical Samples

HBV-induced HCC specimens and nontumor tissues were collected from our hospital and were stored in liquid nitrogen until used. This research was agreed by the Clinical Ethics Committee of The Fourth Hospital of Harbin Medical University and informed consents were obtained.

### 2.2. Cell Transfection and Culture

HCC cells without HBV infection HepG2 and HepG2.2.15 (HCC cell with HBV infection) were purchased from ATCC and cultured in DMEM medium (Gibco, USA), supplemented by streptomycin, penicillin, and FBS. pcDNA-control, pcDNA-TFAP2A-AS1, si-control and si- TFAP2A-AS1, miR-scramble, and miR-933 mimic were synthesized from GenePharma (Shanghai, China). Cell transfection was performed by Lipofectamine2000 with the product's protocol.

### 2.3. Luciferase Reporter Gene Assay

Fragment from 3′UTR of TFAP2A-AS1 and mutant 3′UTR of TFAP2A-AS1 containing miR-933 binding sites were incloned into the psiCHECK2 plasmid (Promega, WI, USA). Scramble or miR-933 mimic and HDAC11 wt-3′UTR and HDAC11 mut-3′UTR and luciferase reporter vector were transfected to cells and the luciferase activity was evaluated with Luciferase Reporter kit (Promega).

The article "Long Noncoding RNA TFAP2A-AS1 Suppressed Hepatitis B Virus Replication by Modulating miR-933/HDAC11" was retracted in 2023. Reasons: unreliable results or conclusions; lack of ethics approval or compliance; concerns about the data; concerns about the peer review.

### 2.4. RT-qPCR

RNA was extracted from specimen or cell using the TRIzol kit (Invitrogen, CA, USA) with the product's instructions. RT-qPCR (Quantitative RT-PCR) was employed to measure mRNA, miRNA, and lncRNA expression with TaKaRa SYBR Green (Dalian, China) on 7500 ABI system (Applied Biosystems, CA, USA). The method of 2^-*ΔΔ*Ct^ was utilized to calculate relative fold change. Primers are shown as follows: GAPDH: F, 5′-TGTTCG TCATGG GTGTGA AC-3′, 5′-ATGGCA TGGACT GTGGTC AT-3′; miR-933: F, 5′-ATTATA TGTGCG CAGGGA GACC-3′, R, 5′-GCGAGC ACAGAA TTAATA CGACTC ACTATA GG-3′; TFAP2A-AS1: F, 5′-CTTGAC AGCTCC AGGGGT TA-3′, R, 5′-TCTAGA CTTGCA GGCACA CA-3′.

### 2.5. HBV Replication and Gene Expression Analysis

The DNA of HBV from cell supernatants was extracted by the Viral Column DNA out reagent (TIANDZ, China) following to the product's information and measured with RT-qPCR method. The HBsAg (hepatitis B surface antigen) and HBeAg (hepatitis B e antigen) expression in supernatants of HCC cell was determined with the ELISA reagent (Biotech, Shanghai).

### 2.6. Statistical Analysis

Data were analyzed with SPSS-19.0 (Chicago, USA) and showed as the mean ± SD (standard deviation). Student's *t*-test was applied to measure comparison difference between two groups. *p* data of <0.05 was represented as significant.

## 3. Results

### 3.1. TFAP2A-AS1 Level in HBV-Associated HCC Samples

RT-qPCR assay was carried out to determine TFAP2A-AS1 in HCC cell, HBV-infected HCC samples, and nontumor tissues. As indicated in Figure 1(a), TFAP2A-AS1 was downregulated in HCC cell lines compared with HL-7702. TFAP2A-AS1 level was lower in HBV-infected HCC samples compared with nontumor tissues (Figure 1(b)). Moreover, TFAP2A-AS1 was downregulated in 31 cases (77.5%) compared to nontumor tissues (Figure 1(c)).

### 3.2. miR-933 Level in HBV-Associated HCC Samples

RT-qPCR analysis was carried out to detect miR-933 expression in HCC cell, HBV-infected HCC samples, and nontumor tissues. As indicated in Figure 2(a), miR-933 was upregulated in HCC cell lines compared to HL-7702. MiR-933 level was higher in HBV-infected HCC samples compared to nontumor tissues (Figure 2(b)). Moreover, miR-933 was upregulated in 27 cases (67.5%) compared to nontumor tissues (Figure 2(c)). MiR-933 expression was negatively associated with TFAP2A-AS1 expression in HBV-correlated HCC samples (Figure 2(d)).

### 3.3. TFAP2A-AS1 Sponged miR-933 in HCC Cell

MiR-933 was significantly upregulated in HepG2.2.15 cell after transfected with miR-933 mimic (Figure 3(a)). Based on the bioinformatics Starbase forecast (http://starbase.sysu.edu.cn/index.php), TFAP2A-AS1 potentially bind to miR-933 (Figure 3(b)). Elevated expression of miR-933 decreased luciferase activity of TFAP2A-AS1-Wt but not TFAP2A-AS1-Mut (Figure 3(c)). RT-qPCR assay showed that TFAP2A-AS1 was overexpressed in HepG2.2.15 cell after transfected with pcDNA-TFAP2A-AS1 (Figure 3(d)). Overexpression of TFAP2A-AS1 repressed miR-933 expression in HepG2.2.15 cell (Figure 3(e)).

The article "Long Noncoding RNA TFAP2A-AS1 Suppressed Hepatitis B Virus Replication by Modulating miR-933/HDAC11" was retracted in 2023. Reasons: unreliable results or conclusions; lack of ethics approval or compliance; concerns about the data; concerns about the peer review.

### 3.4. miR-933 Targeted HDAC11 in HCC Cell

Based on the bioinformatics TargetScan system (http://www.targetscan.org/vert_72/), HDAC11 potentially bind to miR-933 (Figure 4(a)). Overexpression of miR-933 suppressed luciferase activity of HDAC11-Wt but not HDAC11-Mut (Figure 4(b)). RT-qPCR assay was performed and indicated that elevated expression of miR-933 suppressed HDAC11 in HepG2.2.15 cell (Figure 4(c)). Overexpression of HDAC11 promoted HDAC11 expression in HepG2.2.15 cell (Figure 4(d)).

### 3.5. TFAP2A-AS1 and miR-933 Level in HBV-Infected Cell

The levels of TFAP2A-AS1, miR-933, and HDAC11 were detected by qRT-PCR analysis in HBV-infected HepG2 (HepG2.2.15) cell and HepG2 cell. TFAP2A-AS1 expression was downregulated in HepG2.2.15 cell compared to HepG2 cell (Figure 5(a)). MiR-933 level was overexpressed in HepG2.2.15 cell compared to HepG2 cell (Figure 5(b)). Moreover, HDAC11 expression was decreased in HepG2.2.15 cell compared to HepG2 cell (Figure 5(c)).

### 3.6. TFAP2A-AS1 Inhibited HBV Replication and Infection

To identify whether TFAP2A-AS1 regulated HBV replication and expression, cell was treated with pcDNA-control, pcDNA-TFAP2A-AS1, si-control, and si-TFAP2A-AS1, respectively. RT-qPCR assay was carried out to indicate that TFAP2A-AS1 was downregulated in HepG2.2.15 cell after transfected with si-TFAP2A-AS1 (Figure 6(e)). Ectopic expression of TFAP2A-AS1 suppressed cell growth (Figure 6(a)), while TFAP2A-AS1 knockdown enhanced cell proliferation in HepG2.2.15 cell using CCK-8 assays (Figure 6(f)). HbsAg and HbeAg levels were determined with ELISA, and DNA replication of HBV was detected by RT-qPCR. Elevated expression of TFAP2A-AS1 suppressed DNA replication of HBV (Figure 6(b)), while knockdown of TFAP2A-AS1 increased HBV DNA replication (Figure 6(g)). Moreover, TFAP2A-AS1 overexpression inhibited expression of HbsAg (Figure 6(c)) and HbeAg (Figure 6(d)), while TFAP2A-AS1 knockdown enhanced their expression (Figures 6(h) and 6(i)).

### 3.7. miR-933 Increased HBV Replication and Infection

To learn whether miR-933 modulate HBV replication and expression, cell was treated with scramble and miR-933 mimic, respectively. Ectopic expression of miR-933 promoted cell growth in HepG2.2.15 cell using CCK-8 assays (Figure 7(a)). Elevated expression of miR-933 promoted DNA replication of HBV (Figure 7(b)). Ectopic expression of miR-933 enhanced the expression of HbsAg (Figure 7(c)) and HbeAg (Figure 7(d)).

The article "Long Noncoding RNA TFAP2A-AS1 Suppressed Hepatitis B Virus Replication by Modulating miR-933/HDAC11" was retracted in 2023. Reasons: unreliable results or conclusions; lack of ethics approval or compliance; concerns about the data; concerns about the peer review.

### 3.8. TFAP2A-AS1 Suppressed HBV Replication and Infection through Modulating HDAC11

To study whether TFAP2A-AS1 suppressed HBV replication and infection through regulating HDAC11, cells were transfected with si-TFAP2A-AS1 and cotransfected pcDNA-HDAC11 or its pcDNA-control. The results indicated that knockdown of TFAP2A-AS1 enhanced HBV DNA replication, while cotransfection with pcDNA-HDAC11 inhibited HBV DNA replication (Figure 8(a)). Ectopic expression of HDAC11 suppressed the expression of HbeAg (Figure 8(b)) and HbsAg (Figure 8(c)) in TFAP2A-AS1 knockdown-HepG2.2.15 cells.

## 4. Discussion

To improve the treatment of HBV infection and associated HCC, new therapies must be explored. We firstly showed that TFAP2A-AS1 was downregulated in HCC cell lines and HBV-infected HCC samples compared to nontumor tissues. However, miR-933 was upregulated in HCC cell lines and HBV-infected HCC samples compared to nontumor tissues, and miR-933 was negatively associated with the expression of TFAP2A-AS1 in HBV-correlated HCC samples. The expression of TFAP2A-AS1 and HDAC11 was decreased while miR-933 was overexpressed in HBV-infected cell HepG2.2.15. TFAP2A-AS1 acted as one sponge for miR-933 and HDAC11 was one direct target gene for miR-933. Ectopic expression of TFAP2A-AS1 suppressed cell growth, HBV DNA replication, HbeAg, and HbsAg expression, while knockdown of TFAP2A-AS1 enhanced cell proliferation, HBV DNA replication, HbeAg, and HbsAg expression in HepG2.2.15 cell. In addition, ectopic expression of miR-933 promoted cell growth, HBV DNA replication, HbeAg, and HbsAg expression in HepG2.2.15 cell. TFAP2A-AS1 suppressed HBV replication and infection through modulating HDAC11. These data illustrated that TFAP2A-AS1 acted crucial roles in the modulation of HBV replication and may be one potential therapeutic target for HBV infection.

Studies have shown that lncRNAs exerted crucial roles in multiple tumor types and modulated various biological processes [29–31]. For instance, Deng et al. [32] showed that lncRNA F11-AS1 suppressed HBV-associated HCC development through modulating miR-211-5p/NR1I3. Feng et al. indicated that PCNA and lncRNA PCNAP1 was upregulated in HBV-infectious chimeric mice and PCNAP1 promoted HBV replication via regulating PCNA/miR-154/HBV signaling [33]. LncRNA H19 was proved to induce HBV-related HCC development by modulating miR-22 [34]. Recently, TFAP2A-AS1 was identified to be downregulated in breast cancer cell and samples and TFAP2A-AS1 overexpression suppressed cell invasion and proliferation and decreased tumor development in vivo [28]. We also found that TFAP2A-AS1 was downregulated in HCC cell lines and HBV-infected HCC samples. Ectopic expression of TFAP2A-AS1 suppressed cell growth, HBV DNA replication, HbeAg, and HbsAg expression, while knockdown of TFAP2A-AS1 enhanced cell proliferation, HBV DNA replication, HbeAg, and HbsAg expression in HepG2.2.15 cell.

The article "Long Noncoding RNA TFAP2A-AS1 Suppressed Hepatitis B Virus Replication by Modulating miR-933/HDAC11" was retracted in 2023. Reasons: unreliable results or conclusions; lack of ethics approval or compliance; concerns about the data; concerns about the peer review.

Multiple studies have shown that lncRNA participated in tumor progression and occurrence by acting as one sponge for miRNAs and their correlated genes [35–37]. Zhao et al. [38] found that lncRNA TINCR inhibited HCC invasion and growth through sponging miR-218-5p/DDX5. Wu et al. [39] showed that lncRNA SUMO1P3 induced HCC development by promoting Wnt/*β*-catenin pathway via sponging miR-320a. Dai et al. [40] demonstrated that lncRNA TUG1 enhanced HCC progression through modulating DLX2/miR-216b-5p axis. Zheng et al. [41] demonstrated that linc00467 promoted HCC development through sponging NEDD9/miR-18a-5p. A recent study showed that TFAP2A-AS1 suppressed breast cancer progression through sponging miR-933 [28]. Based on the bioinformatics TargetScan system, HDAC11 can potentially bind to miR-933. Overexpression of miR-933 suppressed luciferase activity of HDAC11-Wt but not HDAC11-Mut. Overexpression of TFAP2A-AS1 repressed miR-933 in HepG2.2.15 cell. MiR-933 expression level was higher in HBV-infected HCC samples compared to nontumor tissues. miR-933 expression was negatively associated with the expression of TFAP2A-AS1 in HBV-correlated HCC samples. Moreover, HDAC11 suppressed HBV replication via epigenetic inhibition of cDNA transcription [42]. Furthermore, we showed that TFAP2A-AS1 suppressed HBV replication and infection through modulating HDAC11.

Our manuscript has some limitations. The sample size is small and more samples are needed to study the expression of TFAP2A-AS1. Secondly, the function of TFAP2A-AS1 needs to be verified in vivo.

## 5. Conclusion

Collectively, our data showed that TFAP2A-AS1 was downregulated in HCC cell lines and HBV-infected HCC samples, and ectopic expression of TFAP2A-AS1 suppressed HBV replication and infection through modulating miR-933/HDAC11. These data suggested that TFAP2A-AS1 may be a potential therapeutic target for HBV infection.

## Figures and Tables

**Figure 1:** TFAP2A-AS1 level in HBV-associated HCC samples. (a) TFAP2A-AS1 expression was detected by RT-qPCR assay in HCC cell lines and HL-7702. (b) TFAP2A-AS1 in HBV-infected HCC samples and no-tumor tissues was measured by RT-qPCR analysis. (c) TFAP2A-AS1 was downregulated in 31 cases (77.5%) compared to no-tumor tissues.

The article "Long Noncoding RNA TFAP2A-AS1 Suppressed Hepatitis B Virus Replication by Modulating miR-933/HDAC11" was retracted in 2023. Reasons: unreliable results or conclusions; lack of ethics approval or compliance; concerns about the data; concerns about the peer review.

**Figure 2:** miR-933 level in HBV-associated HCC samples. (a) miR-933 expression was detected by RT-qPCR assay in HCC cell lines and HL-7702. (b) miR-933 in HBV-infected HCC samples and no-tumor tissues was measured by RT-qPCR analysis. (c) miR-933 was upregulated in 27 cases (67.5%) compared to no-tumor tissues. (d) miR-933 was negatively associated with expression of TFAP2A-AS1 in HBV-correlated HCC samples.

**Figure 3:** TFAP2A-AS1 sponged miR-933 in HCC cell. (a) The miR-933 expression was detected by RT-qPCR assay. (b) Based on bioinformatics Starbase forecast (http://starbase.sysu.edu.cn/index.php), TFAP2A-AS1 potentially binded to miR-933. (c) Elevated expression of miR-933 decreased luciferase activity of TFAP2A-AS1-Wt but not TFAP2A-AS1-Mut. (d) RT-qPCR assay was carried out to show that TFAP2A-AS1 was overexpressed in HepG2.2.15 cell after transfected with pcDNA-TFAP2A-AS1. (e) Overexpression of TFAP2A-AS1 repressed miR-933 in HepG2.2.15 cell. ^∗∗^*p* < 0.01.

**Figure 4:** miR-933 targeted HDAC11 in HCC cell. (a) Based on bioinformatics TargetScan system (http://www.targetscan.org/vert_72/), HDAC11 potentially binded to miR-933. (b) Overexpression of miR-933 suppressed luciferase activity of HDAC11-Wt but not HDAC11-Mut. (c) RT-qPCR assay was performed to indicate that elevated expression of miR-933 suppressed HDAC11 in HepG2.2.15 cell. (d) Overexpression of HDAC11 promoted HDAC11 level in HepG2.2.15 cell. ^∗∗^*p* < 0.01.

**Figure 5:** TFAP2A-AS1 and miR-933 level in HBV-infected cell. (a) TFAP2A-AS1 was downregulated in HepG2.2.15 cell compared to HepG2 cell. (b) The miR-933 level was measured by RT-qPCR assay. (c) The miR-933 HDAC11 was measured by RT-qPCR assay.

**Figure 6:** TFAP2A-AS1 inhibited HBV replication and infection. (a) Ectopic expression of TFAP2A-AS1 suppressed cell growth in HepG2.2.15 cell. (b) Elevated expression of TFAP2A-AS1 suppressed DNA replication of HBV. (c) TFAP2A-AS1 overexpression inhibited HbsAg expression in HepG2.2.15 cell. (d) Elevated expression of TFAP2A-AS1 HbeAg expression in HepG2.2.15 cell. (e) The expression of TFAP2A-AS1 was detected by RT-qPCR assay. (f) TFAP2A-AS1 knockdown enhanced cell proliferation in HepG2.2.15 cell using CCK-8 assays. (g) Knockdown of TFAP2A-AS1 increased HBV DNA replication. (h) TFAP2A-AS1 knockdown enhanced HbsAg expression. (i) HbeAg level was determined with ELISA. ^∗^*p* < 0.05, ^∗∗^*p* < 0.01, and ^∗∗∗^*p* < 0.001.

**Figure 7:** miR-933 increased HBV replication and infection. (a) Ectopic expression of miR-933 promoted cell growth in HepG2.2.15 cell using CCK-8 assays. (b) Elevated expression of miR-933 promoted DNA replication of HBV. (c) Ectopic expression of miR-933 enhanced HbsAg expression. (d) HbeAg level was determined with ELISA. ^∗^*p* < 0.05, ^∗∗^*p* < 0.01, and ^∗∗∗^*p* < 0.001.

The article "Long Noncoding RNA TFAP2A-AS1 Suppressed Hepatitis B Virus Replication by Modulating miR-933/HDAC11" was retracted in 2023. Reasons: unreliable results or conclusions; lack of ethics approval or compliance; concerns about the data; concerns about the peer review.

**Figure 8:** TFAP2A-AS1 suppressed HBV replication and infection through modulating HDAC11. (a) Knockdown of TFAP2A-AS1 enhanced HBV DNA replication, while cotransfection with pcDNA-HDAC11 inhibited HBV DNA replication. (b) HbeAg level was determined with ELISA. (c) HbsAg level was determined with ELISA. ^∗^*p* < 0.05 and ^∗∗^*p* < 0.01.

## Data Availability

The authors can make data available on request through an email to the corresponding author, Lei Yu, Email: widedoor@sina.com and Liying Zhu, Email: zlyhmu@163.com

## Abbreviations

HBV: Hepatitis B virus
HCC: Hepatocellular carcinoma
lncRNAs: Long noncoding RNAs
ncRNAs: Noncoding RNAs
miR-933: microRNA-933
ATCC: American Type Culture Collection
FBS: Fetal bovine serum
cDNAs: Complementary DNAs.
